The article "Euryops arabicus Promotes Healing of Excised Wounds in Rat Skin: Emphasis on Its Collagen-Enhancing, Antioxidant, and Anti-Inflammatory Activities" was retracted in 2023. Reasons: suspected computer-generated content; unreliable results or conclusions; concerns about the data; concerns about the results or conclusions.

# *Euryops arabicus* Promotes Healing of Excised Wounds in Rat Skin: Emphasis on Its Collagen-Enhancing, Antioxidant, and Anti-Inflammatory Activities

**DOI:** 10.1155/2021/8891445

**Published:** 2021-01-26

**Authors:** Ahmed Abdel-Lateff, Ashraf B. Abdel-Naim, Walied M. Alarif, Mardi M. Algandaby, Najla A. Alburae, Ali M. Alghamdi, Mohammed Z. Nasrullah, Usama A. Fahmy

**Affiliations:** ^1^Department of Natural Products and Alternative Medicine, Faculty of Pharmacy, King Abdulaziz University, Jeddah 21589, P.O. Box 80260, Saudi Arabia; ^2^Department of Pharmacognosy, Faculty of Pharmacy, Minia University, Minia 61519, P.O. Box 61511, Egypt; ^3^Department of Pharmacology and Toxicology, Faculty of Pharmacy, King Abdulaziz University, Jeddah 21589, P.O. Box 80260, Saudi Arabia; ^4^Department of Marine Chemistry, Faculty of Marine Sciences, King Abdulaziz University, Jeddah 21589, P.O. Box 80207, Saudi Arabia; ^5^Department of Biological Sciences, Faculty of Science, King Abdulaziz University, Jeddah 21589, P.O. Box 80203, Saudi Arabia; ^6^Pharmacy Department, Mental Health Hospital, Taif, P.O. Box 2056, Saudi Arabia; ^7^Center of Excellence for Drug Research and Pharmaceutical Industries, King Abdulaziz University, Jeddah 21589, Saudi Arabia; ^8^Mohamed Saeed Tamer Chair for Pharmaceutical Industries, King Abdulaziz University, Jeddah 21589, Saudi Arabia; ^9^Department of Pharmaceutics, Faculty of Pharmacy, King Abdulaziz University, Jeddah 21589, Saudi Arabia

## Abstract

*Euryops arabicus* Steud (*E. arabicus*) belongs to the family Asteraceae. It has several uses in folk medicine in the Arabian Peninsula. The current study aimed at evaluating the wound healing properties of the *E. arabicus* extract in rats. Primarily, *E. arabicus* successfully accelerated cell migration *in vitro* and it also showed no signs of dermal toxicity. Topical application of *E. arabicus* extract (5% or 20%) expedited healing of excised skin in rats. Histological examinations indicated that *E. arabicus* shortened epithelization period, stimulated fibroblast activity, and increased collagen deposition in wound tissues. The plant extract exerted antioxidant activity as evidenced by inhibition of GSH depletion and MDA accumulation and enhanced mRNA expression of Sod1 in wound tissues collected at the end of the experiment. Further, *E. arabicus* inhibited the rise of TNF-*α* and IL-1*β* in the skin wound region. The anti-inflammatory was confirmed by the observed down regulation of Ptgs2, Nos2, IL-6, and NF-*κ*B mRNA expression. In addition, the extract enhanced the expression of TGF-*β*1 and HIF-1*α* in wounded skin tissues as indicated immunohistochemically. Conclusively, *E. arabicus* expedites excision wound healing in rats. Collagen-enhancing, anti-inflammatory, and antioxidant properties mediate the observed wound healing activity. These findings might contribute to our understanding of the ethnobotanical use of *E. arabicus* in wounds.

## 1. Introduction

Wound is an outcome of physical trauma, which results from any agent that causes cutting, puncture, or contusion in the skin. It ranges from simple abrasion to serious avulsion. The skin has two main layers: epidermis and dermis. They exist in a steady state of equilibrium, forming an external protective barrier [1]. Wounds lead to inflammatory proliferation, which affects normal structure, function, and architecture of the skin [2]. Wound healing is a complex process of repairing the damaged tissues. It includes several phases: hemostasis, inflammation, epithelialization, and maturation [3]. Unluckily, delayed closure of a wound has a significant influence on the quality of patients' life. It leads to loss of function and mobility; anxiety, distress, and social withdrawal; extended hospital stays; and chronic morbidity [4–7]. Therefore, wound dressings'materials have witnessed continuous advancements and improvements [8].

Members of the family Asteraceae are ubiquitous throughout the world with 1900 genera and 32,000 species. It is the largest plant family of flowering plants. Several Asteraceae plants are used in human diets and remedies along with garden ornamentals. *E. arabicus* Steud is a plant that belongs to the family Asteraceae. It is one of the traditional medicinal plants used widely in the Arabian Peninsula especially the southwestern region. It has been used in folk medicine for several diseases that include pain, inflammation, and skin injuries [9–11]. It has been reported that *E. arabicus* has essential oils [12], terpenoids [13], and flavonoids [12, 13]. In addition, *E. arabicus* has proven to possess antioxidant, antimicrobial, hepatoprotective, and anti-inflammatory activities [9, 12, 14, 15].

Therefore, the current work was designed to explore the potential effect of *E. arabicus* extract to accelerate excision wound healing in rats.

## 2. Materials and Methods

### 2.1. Assessment of Acute Dermal Toxicity

Acute dermal toxicity of *E. arabicus* extract was determined using a limit dose of 2000 mg/kg in 5 male rats and repeated in additional 5 rats. Approximately 24 h before the experiment, fur was removed from the dorsal area of the trunk by careful shaving. The saved areas were about 10% of the total body surface area of each rat. The limit dose was prepared in Vaseline (white petrolatum, Unilever, London, UK) (1 g *E. arabicus* extract : 1 g Vaseline) and applied to the shaved areas. Animals were observed for 14 days giving special attention during the first 24 h. The procedure complies with OECD guideline for testing of chemicals no. 434 (OECD, 2004) [16].

### 2.2. Plant Material

The aerial parts of *E. arabicus* Steud (Asteraceae) were collected from Al-Taif, Saudi Arabia (21°03′00.0^″^N 43°23′00.0^″^E), in February 2019. A sample (Feb-20-EA-1) was kept in the herbarium of Faculty Pharmacy, KAU, Jeddah, Saudi Arabia.

### 2.3. Extraction

The extraction process has been applied as previously reported [9]. The powdered air-dried aerial parts of *E. arabicus* (400 g) were extracted twice with mixture of CHCl_3_ : MeOH (1 : 1, 15 L X 3) at 20–23°C for a week, and then, the combined extracts were concentrated till drying, under reduced pressure, using rotary evaporator, to obtain (38 g, 9.5 % yield) blackish gummy residue.

### 2.4. Chemical Investigation of Extract of *E. arabicus*

Chemical investigation of the extract of *E. arabicus* resulted in the identification of five flavonoidal compounds. Five methoxyflavonol derivatives were previously identified as 5-hydroxy-4′,6,7,8-tetramethoxyflavone, 5-hydroxy-3′,4′,6,7,8-pentamethoxy flavone, 5-hydroxy-3′,4′,6,7-tetramethoxyflavone, 5,5′-dihydroxy-3′,4′,6,7-tetramethoxy flavone, and 5,8-dihydroxy-3′,4′,6,7-tetramethoxyflavone [9].

### 2.5. Determination of IC_50_ of *E. arabicus* Extract in Human Neonatal Foreskin Epidermal Keratinocyte (HEK) Cells and In Vitro Cell Migration Assay

Human neonatal foreskin epidermal keratinocytes (HEK) were purchased from Modern Tissue Technologies Inc. (Seoul, Korea). HEK was grown on Dermal Cell Basal Medium (Bioz, Los Altos, CA, USA) containing 10% fetal bovine serum, penicillin (100 IU/ml), and streptomycin (100 mg/ml) at 37°C in a humidified atmosphere containing 5% CO_2_. IC_50_ was determined using an MTT assay kit (Sigma-Aldrich, St. Louis, MO, USA). Also, a migration assay was performed using CytoSelect™ 24-Well Wound Healing Assay (Cell Biolabs, Inc., San Diego, CA, USA). Inserts were placed in the plate wells with their wound field aligned in the same direction. Cells (5 × 10^5^ cells/well) were added to each well by inserting the pipette tip through the opening end at the top of the insert. Cells were incubated for 24 h until a monolayer formed. Inserts were then removed from the well, and the media were discarded. Various concentrations of *E. arabicus* and media were added to the wells. Cells were incubated for 48 h. The migration rate of the cells was measured in the wound field via assessing wound width.

### 2.6. Preparation of *E. arabicus* in Vaseline

A topical ointment of the *E. arabicus* extract was prepared by using the incorporation method. Dried *E. arabicus* extract (5 g) was powdered and blended with 10 g Vaseline in a mortar. Vaseline then was added potion wise and blended till 100 g (for 5% *w*/*w*). Another concentration was achieved by mixing the dried *E. arabicus* extract (20 g) with 40 g Vaseline in a mortar. Vaseline then was added potion wise and blended till 100 g (for 20% *w*/*w*). The choice of *E. arabicus* concentrations was based on a preliminary experiment.

### 2.7. Animals

Fifty male Wistar rats (200-230 g) were obtained from the animal facility, King Abdulaziz University (KAU). Animals were kept on a 12 h light-dark cycle and a temperature of 22 ± 2°C. The Committee of Research Ethics, Faculty of Pharmacy, KAU, approved all animal handling procedures (Reference # PH-126-41).

### 2.8. Excision Wounding and Animal Treatment

Rats were anesthetized by an intraperitoneal injection of ketamine (100 mg/kg)/xylazine (10 mg/kg). Then, the dorsal surface was shaved and the exposed skin was sterilized with 70% ethanol. Afterwards, a full-thickness excision circle of 1 cm in diameter was made on rats' dorsal surface. Then, wounds were disinfected after the excision was completed. Lidocaine hydrochloride (2%) containing 1 : 80,000 epinephrine (4.4 mg/kg) was injected subcutaneously close to the wound area directly after wounding to reduce pain.

Wounded rats were organized in 5 groups (10 each): group 1: untreated control rats with no treatment; group 2: negative control rats received treated topical daily Vaseline ointment (0.5 g) in the wound area; group 3: positive control rats treated with 0.5 g of Mebo® ointment [17], Julfar UE (𝛽-sitosterol, baicalin, and berberine as active ingredients in a base of beeswax and sesame oil) in the wound area; group 4: Vaseline ointment preparation of *E. arabicus* (5% *w*/*w*); and group 5: Vaseline ointment preparation of *E. arabicus* (20% *w*/*w*).

All treatments were applied topically every day for 14 days. Then, wounds were covered with Vaseline gauze dressings and changed once daily. Wounds were measured and photographed on 0, 3, 7, 10, and 14 days. At day 7, 4 animals from each group were sacrificed by ether overdose and the skin in the wound area was dissected out and kept in 10% neutral formalin. On day 14, the rest of the animals in all groups were sacrificed by ether overdose and the skin in the wound area was dissected out. Part of the skin from each animal was kept in 10% neutral formalin, and the other part was kept in -80°C for further analyses.

### 2.9. Wound Measurement

Wound contraction percentage was calculated by utilizing the following formula:

(1) $$\begin{array}{c} \text{Wound contraction}\%=\frac{\text{Day zero wound diameter}-\text{Day }14\text{ wound diameter}}{\text{Day zero wound diameter}}\times 100. \end{array}$$

### 2.10. Preparation of Tissue Homogenate

Tissues were carefully rinsed with ice-cooled saline, gently blotted between filter papers, and weighed. Ten percent of homogenates were prepared in ice-cold phosphate-buffered saline (50 mM potassium phosphate, pH 7.4) at 4°C. Homogenates were used for subsequent biochemical analyses.

### 2.11. Histological Examination

Wound tissues collected on days 7 and 10 were kept in neutral formalin (10%) for 24 h. This was followed by dehydration in serial concentrations of ethanol, cleared in xylene, and inserted in paraffin. Tissues in paraffin block were sectioned (5 *μ*m thickness). After dewaxing, tissues were rehydrated. Some sections were stained using H&E, and the rest were stained with Masson's trichrome. Histological examinations were examined by a pathologist without prior knowledge of the treatment groups. Based on the degree of reepithelization, fibroblast proliferation, collagen deposition, inflammatory cell infiltration, and wound healing phase (I, II, or III) on day 7 were given score based on their abundance ranging from − to +++.

### 2.12. Biochemical Analyses

Malondialdehyde (MDA), reduced glutathione (GSH), and protein concentration were determined using commercially available kits (Biodiagnostic, Cairo, Egypt). Tumor necrosis factor-*α* (TNF-*α*) and interleukin-1*β* (IL-1*β*) were estimated using rat ELISA kits obtained from Elabscience, Houston, TX, USA.

### 2.13. RT-qPCR in Excised (Healing/Healed) Tissue

Tissues from each rat on day 14 were homogenized in an ultrasonic probe. RNA was extracted utilizing a nucleic acid extraction kit (NucleoSpin®) purchased from Macherey-Nagel GmbH & Co. KG, Duerin, Germany. Purity (A260/A280 ratio) and concentration of RNA were determined using spectrophotometric analyses (dual-wavelength Beckman spectrophotometer, USA). Reverse transcription and real-time PCR was undertaken using SensiFAST™ SYBR® Hi-ROX One-Step Kit, Cat. No. BIO-73005 (Bioline, a Meridian Bioscience company, London, UK). PCR amplification reactions were then performed using the following primers purchased from Qiagen, Valencia, CA, USA: Sod1 (QT00174888), Ptgs2 (QT00192934), Nos2 (QT00178325), IL-6 (PPR06483B), and NF-*κ*B (QT00370545) and the housekeeping gene GAPDH (QT00199633), using StepOne Real-Time PCR System (Applied Biosystems, Foster City, CA, USA). The relative quantitation (RQ) of the assessed genes to GAPDH was determined according to the calculation of delta-delta Ct (*ΔΔ*Ct).

### 2.14. Immunohistochemical Analyses

Skin tissue sections were dried using autoclave, deparaffinized, and rehydrated using ethanol. Then, they were boiled in citrate buffer (pH 6.0) for ten minutes. Afterwards, the sections were incubated in 5% bovine serum albumin (BSA) in tris-buffered saline (TBS) for two hours followed by immersion overnight at 4°C with the primary antibodies (1 *μ*g/ml). These were rabbit monoclonal anti-TGF beta 1 antibody (catalog # ab215715) and rabbit monoclonal anti-HIF-1 alpha antibody (catalog # ab179483). TBS was used to flush the slides which were then incubated with the biotinylated secondary antibody using a Cell and Tissue Staining Kit (anti-rabbit HPRD-DAB system, catalog # CTS005, R&D Systems, MN, USA). Image analysis was performed for at least three sections per rat, recorded, and quantified by ImageJ analysis software (ImageJ, 1.46a, NIH, USA).

### 2.15. Statistical Analysis

Data are demonstrated as mean ± SD. Multiple comparisons were made using one-way ANOVA followed by Tukey's test. All analyses were performed using GraphPad Prism software®, version 8.0 (GraphPad, La Jolla, CA, USA). The level of *p* < 0.05 was accepted to the criterion of significance.

## 3. Results and Discussion

### 3.1. Cytotoxicity of *E. arabicus*

The data in Figure 1 indicate that the extract is relatively safe to HEK cells with a high IC_50_ value of 385.3 ± 21.2 *μ*g/ml.

### 3.2. *In Vitro* Cell Migration

The percentage of migration of keratinocytes was expressed as a percentage relative to the control group. The distance of cell migration in the treatment groups was reported at 48 h after starting incubation. The distance of cell migration increased significantly in a concentration-related manner (Figure 2).

### 3.3. Acute Dermal Toxicity

A dose limit of 2000 mg/kg of *E. arabicus* extract was applied locally to the shaved skin areas of 5 animals. At 24 h after application, no deaths or evident toxicities were observed. Therefore, the same procedure was repeated using 5 additional animals. Again, no deaths or evident toxicities were detected. Observations of all animals were extended to day 14 and confirmed absence of any evident toxicities. Therefore, the extract is classified as category 5 or unclassified according to the OECD guidelines [16].

### 3.4. Assessment of Wound Healing

Local application of *E. arabicus* extract (5 and 20% *w*/*w*) showed no significant alteration in the rate of wounds till day 7. However, on day 10, *E. arabicus* extract expedited wound healing as compared to the untreated and negative control groups. On day 14, wounds exposed to *E. arabicus* extract (20% *w*/*w*) showed almost complete healing. It is noteworthy to report that the lower concentration of *E. arabicus* extract (5%) showed superior healing activities as compared to the positive control group (Figure 3(a)). Assessment of wound contraction percentage indicated that animals treated with *E. arabicus* extract exhibited significantly higher wound contractions in a dose-related manner (Figure 3(b)).

### 3.5. Histopathological Investigation

#### 3.5.1. Microscopic Examination of Wound Tissues on Day 7 Stained with Hematoxylin and Eosin (H&E)

Wounded skin in animals of the untreated, negative, and positive controls as well as *E. arabicus* (5%) groups showed marked edema and inflammatory infiltrate, which contained neutrophils and macrophages. Proliferating thin-walled and dilated congested blood vessels were also observed. Wounded skin in animals of the *E. arabicus* (20%) group exhibited mild inflammatory infiltrate that contained mainly macrophages and excess thick collagen (Figure 4(a)).

#### 3.5.2. Microscopic Examination of Wound Tissues on Day 7 Stained with Masson's Trichrome (MT)

Sections obtained from the wounded skin in animals of the untreated and negative control groups showed immature thick collagen bundles. However, the positive control and *E. arabicus* (5% and 20%) groups showed excess thin collagen (Figure 4(b)).

#### 3.5.3. Microscopic Examination of Wound Tissues on Day 14 Stained with Hematoxylin and Eosin (H&E)

The wounded skin in animals of the untreated and negative control groups showed moderate edema, and inflammatory infiltrate, which contains macrophages. Proliferating thin-walled and dilated congested blood vessels covered by poorly epithelialized crust were also observed. Wounded skin in animals of the positive control and *E. arabicus* (5%) groups exhibited mild inflammatory infiltrate which contained macrophages and covered by poorly epithelialized crust were observed. Wounded skin in animals of the *E. arabicus* (20%) group showed inflammatory infiltrate which contained macrophages. Proliferating thin-walled and almost normal blood vessels were covered by poorly epithelialized crust (Figure 4(c)).

#### 3.5.4. Microscopic Examination of Wound Tissues on Day 14 Stained with Masson's Trichrome (MT)

Sections obtained from wounded skin in animals of the untreated and negative control groups showed immature thick collagen bundles. However, the positive control and *E. arabicus* (5% or 20%) groups showed excess thin collagen. In addition, the three latter groups exhibited mild vacuolar changes in basal keratinocytes of the epidermis and complete reepithelialization. Further, animals in the *E. arabicus* 20% group showed frequent mature collagen fibers together with hair follicles and less fibrous granulation tissue (Figure 4(d)). Histological features are semiquantitated with regard to reepithelialization, fibroblast proliferation, and collagen deposition as well as different phases of wound healing. It was evident that sections obtained from *E. arabicus* (5% and 20%)-treated animals showed accelerated healing as evidenced by higher portions of skin tissues in phases II and III as compared to untreated controls (Table 1).

#### 3.5.5. Effect of *E. arabicus* on Oxidative Status on Day 14

The data in Figures 5(a) and (b) indicate that wound tissues from animals in the positive control group as well as those treated with *E. arabicus* (5 and 20%) showed significantly lower content of MDA 2.43- and 1.65-fold compared to the untreated and negative control groups. In addition, *E. arabicus* (5%) significantly enhanced GSH in wound tissues by 1.33- and 1.1.64-fold compared to the negative group. *E. arabicus* (5% or 20%) significantly enhanced mRNA expression of Sod1, by almost 3.8-fold increase as the untreated control group (Figure 5(c)).

#### 3.5.6. Effect of *E. arabicus* on TNF-*α* and IL-1*β* on Day 14

Figure 6(a) indicates that *E. arabicus* (5% or 20%) significantly decreased IL-1*β* content in wound tissues to almost 50% of the untreated control values. Similarly, wound tissue content of TNF-*α* was significantly decreased by *E. arabicus* (5% or 20%) by almost 64% and 75% untreated control value on days 7 and 14, respectively (Figure 6(b)). It is noteworthy to report that, effects of *E. arabicus* (5% or 20%) on TNF-*α* and IL-1*β* were comparable to those of the positive control preparation.

#### 3.5.7. Effect of *E. arabicus* on mRNA Expression of Ptgs2, Nos2, IL-6, and NF-*κ*B on Day 14

Figure 7(a) indicates that *E. arabicus* (5% and 20%) significantly down regulated expression of Ptgs2 mRNA approximately 61.0 and 48.4%, to the negative control, respectively. *E. arabicus* (5% and 20%) significantly downregulated the expression of Nos2 mRNA approximately 65.8% and 51.0%, to the negative control, respectively (Figure 7(b)). *E. arabicus* (5% and 20%) significantly downregulated the expression of IL-6 mRNA approximately 38.9% and 31.3%, to the negative control, respectively (Figure 7(c)). *E. arabicus* (5% and 20%) significantly downregulated the expression of NF-*κ*B mRNA approximately 54.6% and 49.4%, to the negative control, respectively (Figure 7(d)).

### 3.6. Assessment of TGF-*β*1 and HIF-1*α* Expression Immunohistochemically

The data in Figure 8 indicate that experimental skin tissues from untreated and negative control animals showed relatively lower expression of both TGF-*β*1 and HIF-1*α*. However, topical application of *E. arabicus* in concentrations of 5 and 20% resulted in significant increase of TGF-*β*1 by 37% and 77% as compared to the negative control group, respectively. Similarly, *E. arabicus* ointment (5% and 20%) boosted HIF-1*α* expression by 26 and 84% as compared to negative control animals. It is noteworthy to report that the higher concentration of the preparation exhibited expression levels of TGF-*β*1 and HIF-1*α* higher than those observed in the positive control-treated rats.

## 4. Discussion

The current investigation was designed to evaluate the potential wound healing properties of *E. arabicus* extract in rats. In the current study, the potential of the extract to expedite wound healing was confirmed by acceleration the migration of the human neonatal foreskin epidermal keratinocytes (HEK) in an *in vitro* assay. *E. arabicus* showed no signs of dermal toxicity and thus can be labelled as class 5 or unclassified according to the OECD guidelines. Our data indicated that topical application of *E. arabicus* (5% *w*/*w*) expedited wound healing, starting on day 10, as compared to the untreated and negative control groups. *E. arabicus* extract (20% *w*/*w*) showed almost complete healing on day 14. It is noteworthy to report that *E. arabicus* extract (5%) showed potent healing effects comparable to the commercially available positive control. This effect may be due to the flavonoidal content of *E. arabicus*. Based on the observation that medicinally active natural compounds facilitate the wound healing process, flavonoids, terpenoids, and essential oils which are major constituents in *E. arabicus* have played a pivotal role in conducting wound healing. Flavonoids showed antiseptic and antimicrobial properties; moreover, the antioxidant effects exerted by most phenolic compounds (including flavonoids) promote the process of wound healing. Essential oils and terpenoids (mostly hydrophobic) are easily absorbed by the skins which help modulate one or more steps of wound healing process [7, 9]. In addition, our observations are consistent with the reported results of different plants [18, 19] with related phytochemical constituents that belong to different chemical classes, including essential oils, flavonoids, terpenoids, and phenolic compounds [20].

Wound healing properties of *E. arabicus* were confirmed by histological examinations of tissues collected at the end of the experiment. *E. arabicus* shortened the epithelization period. Treated animals showed tissues at the remodeling stage with enhanced deposition of collagen at phases II and II of wound healing. In particular, granulation, collagen maturation, and scar formation were frequently seen all over tissue sections. The inflammatory phase has an important role in wound curing. It is characterized by hemostasis and inflammation, whereas epithelization and collagen deposition mark the proliferative phase [21–23]. The observed shortening of the inflammation phase in treated animals is consistent with the reported anti-inflammatory properties of *E. arabicus* [9]. Fibroblasts, collagen, edema, and angiogenesis are the main markers of the wound granulation [19]. This is in addition to collagen deposition which is a crucial step that follows fibroblast activation [24]. Masson's trichrome staining of sections obtained from *E. arabicus*-treated animals confirmed collagen deposition and enhanced angiogenesis.

In the current study, *E. arabicus* exhibited prominent antioxidant activity as evidenced by decreased lipid peroxidation, enhanced glutathione content, and upregulation of Sod1 mRNA expression in wound tissues collected on day 14. This is consistent with previous studies. Five methoxyflavonols with antioxidant, anti-inflammatory, and antichemotactic properties were previously isolated from the plant [9]. MDA designates the occurrence of oxidative stress due to the peroxidation of lipid membranes [25]. Lipid peroxidation can be inhibited by flavonoids, which play a role in enhancing viability of collagen and preventing cell membrane damage [26]. GSH is an endogenous antioxidant and plays a major role in detoxifying free oxidizing radicals [27]. Thus, it indirectly participates in speeding up healing. This is in line with previous reports highlighting the ability of endogenous antioxidants to accelerate all phases of healing [28].

In this investigation, *E. arabicus* showed strong anti-inflammatory effect as it inhibited IL-1*β* and TNF-*α* content in wound tissues. Proinflammatory cytokines such as IL-1*β* and TNF-*α* are enhanced during the inflammatory phase of wound healing. This is a consequence of NF-*κ*B translocation which eventually enhances inflammation and recruitment of neutrophils and macrophages [29]. Also, these events are associated with generation of oxidative stress that has a role in the pathogenesis of wounds. It has been shown that elevated release of TNF-*α* and IL-1*β* causes diminished fibroblast proliferation resulting in delay of wound healing [30]. Also, TNF-*α* inhibits collagen deposition in vivo. In the current work, *E. arabicus* suppressed mRNA expression of NF-*κ*B in wound tissues and decreased production of the proinflammatory mediators TNF-*α* and IL-1*β*. The anti-inflammatory activities were further confirmed by the observed downregulation of Ptgs2, Nos2, IL-6, and NF-*κ*B mRNA expression. These data are supported by previous reports highlighting the anti-inflammatory properties of *E. arabicus* [9], in which markers of inflammation were promptly inhibited in an *in vitro* model of inflammation using peripheral blood mononuclear cells (PBNCs) challenged with carrageenan. However, our data indicated that healing rate differences between treatment groups were pronounced staring only on day 10 and onwards. This suggests that completion of healing is a consequence of passing the inflammation phase. This is in harmony with the notion that the greatest decline in IL-1*β* and TNF-*α* content was observed on day 14. In addition, our data indicate that *E. arabicus* enhanced expression of TGF-*β*1 and HIF-1*α*. Actually, TGF-*β*1 is a central mediator of fibroblast proliferation and repair [31]. This adds additional explanation of the observed wound healing activity of the extract. HIF-1*α* is a regulator of angiogenesis and consequently expedites skin healing [32]. This is consistent with the previously observed formation of blood vessels in our histological studies.

## 5. Conclusions

*E. arabicus* enhances excision wound healing in rats. This can be attributed, at least partly, to its collagen-enhancing, antioxidant, and anti-inflammatory activities. These findings help to understand the ethnic use of the plant for several types of wounds. In the near future, the phytochemical profile of the extract will be studied with the aim of isolation and characterization of active constituents responsible for wound healing properties.

## Figures and Tables

**Figure 1:** IC_50_ of *E. arabicus* in human neonatal foreskin epidermal keratinocyte (HEK) cells.

**Figure 2:** Effect of *E. arabicus* on keratinocyte migration: (a) control, (b) *E. arabicus* (10 *μ*g/ml), (c) *E. arabicus* (100 *μ*g/ml), and (d) *E. arabicus* (1000 *μ*g/ml). Values are given as mean ± SD (*n* = 6). ^a^Significantly different from control at *p* < 0.05.

**Figure 3:** (a) Photographs showing impact of topical *E. arabicus* (5% and 20%) on closure of excision wounds in rats on day 7 and day 14. Scale bar = 0.25 cm. (b) Effects of different treatments on percent wound contraction on day 10 and day 14 in rats. Values are given as mean ± SD (*n* = 6). ^a^Significantly different from untreated control at *p* < 0.05. ^b^Significantly different from negative control at *p* < 0.05.

**Figure 4:** Histopathological effects of *E. arabicus* (5% and 20%) on wound healing on day 7 and day 14. Hematoxylin and eosin (H&E; 100x). Masson's trichrome (MT 400x).

**Figure 5:** Impact of *E. arabicus* (5% and 20%) on (a) MDA, (b) GSH, and (c) mRNA expression of Sod1 in the wound tissues. Values are given as mean ± SD (*n* = 6). ^a^Significantly different from untreated control at *p* < 0.05. ^b^Significantly different from negative control at *p* < 0.05.

**Figure 6:** Effect of *E. arabicus* (5% and 20%) on (a) IL-1*β* and (b) TNF-*α* in the wound tissues on days 7 and 14. Values are given as mean ± SD (*n* = 6). ^a^Significantly different from untreated control at *p* < 0.05. ^b^Significantly different from negative control at *p* < 0.05.

**Figure 7:** Effect of *E. arabicus* (5% and 20%) on mRNA expression of (a) Ptgs2, (b) Nos2, (c) IL-6, and (d) NF-*κ*B in wound tissue. Data are expressed as mean ± SD (*n* = 6). ^a^Significantly different from untreated control at *p* < 0.05. ^b^Significantly different from negative control at *p* < 0.05.

**Figure 8:** Effect of *E. arabicus* on expression of TGF-*β*1 and HIF-1*α* in wound tissues of rats. Values are given as mean ± SD (*n* = 6). ^a^Significantly different from untreated control at *p* < 0.05. ^b^Significantly different from negative control at *p* < 0.05. ^c^Significantly different from positive control at *p* < 0.05. ^d^Significantly different from *E. arabicus* 5% at *p* < 0.05.

**Table 1:** Histological features of wound healing in animals treated topically with *E. arabicus* on day 7.

	RE	FP	CD	IC	Phase I	Phase II	Phase III
Untreated control	−	++	++	++	++	++	−
Negative control	−	++	+	++	++	++	−
Positive control	+	+	++	+	+	+++	++
*E. arabicus* (5%)	−	+/−	+	+	+	++	+
*E. arabicus* (20%)	+	+	++	+/−	+	+++	++

RE = reepithelization; FP = fibroblast proliferation; CD = collagen deposition; IC = inflammatory cell infiltration; phase I = inflammation phase of wound healing; phase II = proliferation phase of wound healing; phase III = remodeling phase of wound healing (−, +, ++, and +++ refer to nil, low, moderate, and highly abundant).

## Data Availability

We inserted all obtained data and results in the uploaded version of our manuscript.
